The article "Aerial Separation and Receiver Arrangements on Identifying Lung Syndromes Using the Artificial Neural Network" was published in 2022. Journal: Comput Intell Neurosci.

# Aerial Separation and Receiver Arrangements on Identifying Lung Syndromes Using the Artificial Neural Network

**DOI:** 10.1155/2022/7298903

**Published:** 2022-08-23

**Authors:** Hariprasath Manoharan, Radha Krishna Rambola, Pravin R. Kshirsagar, Prasun Chakrabarti, Jarallah Alqahtani, Quadri Noorulhasan Naveed, Saiful Islam, Walelign Dinku Mekuriyaw

**Affiliations:** ^1^Department of Electronics and Communication Engineering, Panimalar Engineering College, Poonamallee, Chennai, India; ^2^Department of Computer Science and Engineering, SVKM's NMIMS MPSTME Shirpur Campus, Dhule, India; ^3^Department of Artificial Intelligence, G. H. Raisoni College of Engineering, Nagpur, India; ^4^Deputy Provost, ITM SLS Baroda University, Vadodara, India; ^5^College of Computer Science and Information Systems, Najran University, Najran 61441, Saudi Arabia; ^6^College of Computer Science, King Khalid University, Abha 61413, Saudi Arabia; ^7^Civil Engineering Department, College of Engineering, King Khalid University, Abha 61421, Asir, Saudi Arabia; ^8^Department of Chemical Engineering, College of Biological and Chemical Engineering, Addis Ababa, Ethiopia

## Abstract

Lung disease is one of the most harmful diseases in traditional days and is the same nowadays. Early detection is one of the most crucial ways to prevent a human from developing these types of diseases. Many researchers are involved in finding various techniques for predicting the accuracy of the diseases. On the basis of the machine learning algorithm, it was not possible to predict the better accuracy when compared to the deep learning technique; this work has proposed enhanced artificial neural network approaches for the accuracy of lung diseases. Here, the discrete Fourier transform and the Burg auto-regression techniques are used for extracting the computed tomography (CT) scan images, and feature reduction takes place by using principle component analysis (PCA). This proposed work has used the 120 subjective datasets from public landmarks with and without lung diseases. The given dataset is trained by using an enhanced artificial neural network (ANN). The preprocessing techniques are handled by using a Gaussian filter; thus, our proposed approach provides enhanced classification accuracy. Finally, our proposed method is compared with the existing machine learning approach based on its accuracy.

## 1. Introduction

Lung disease is one of the major diseases nowadays, so the early detection and prevention of the disease are more crucial; many researchers are involved to create more and more algorithms in detecting the accuracy of lung disease classifications. In simple words, lung diseases are considered a disorder that arises from different categories, and then the various types of diseases are found in the lung disease classifications, namely, asthma, COPD, infections like influenza, pneumonia, and tuberculosis, lung cancer, and many other breathing problems. The most common types of lung cancer are lung nodules, non-small-cell lung cancer, and mesothelioma. There are two types of lung cancer, namely, small cell lung cancer and non-small cell lung cancer [1–3].

The article "Aerial Separation and Receiver Arrangements on Identifying Lung Syndromes Using the Artificial Neural Network" was published in 2022. Journal: Comput Intell Neurosci.

Non-small-cell lung cancer is further divided into three types, and these are all considered the normal form of the disease; thus, the carcinoma type has various types, namely, large cell carcinoma and squamous cell carcinoma; and adenocarcinoma is the most common lung cancer that is found all over the world. The Internet of Things plays a vital role in lung disease classifications and the artificial intelligence protocol plays an important role in the form of cell diseases. The researcher used the form of the support vector machine, the fuzzy-based clustering, and the *K* nearest neighbor technique to predict the better accuracy of the diseases, but it could not produce a better accuracy of the classifications. Thus, our paper implements an artificial neural network for the classification of the given datasets, and the feature extraction is detected by using particle swarm optimization. Artificial neural networks (ANNs) are statistical models that simulate the learning dynamics of the brain by replicating the biological organization of neural cells through a mathematical structure. Although there may be a variety of definitions for the term “ANN,” it typically refers to a neural network used for modeling nonlinear statistical data. The neural models used today in a variety of medical specialties, including oncology, are effective models for nonlinear regression or classification and do not seek to be physiologically realistic in every detail. Applications for ANN inference exist in tasks that demand attention and focus. The success of ANNs in clinical decision support depends critically on better integration with clinical protocols, awareness of the necessity of combining various paradigms to produce the overall reasoning structure that is the simplest and most transparent, and the willingness to test this in a real clinical setting. We have evaluated the evidence supporting advancements in the application of ANN in lung cancer research [4–14].

### 1.1. Review of Literature

Sathawane et al. [15] have implemented the convolutional neural network for biomedical applications in health care. The image processing in the medical field has been used for getting better accuracy and processing time in the entire datasets; thus, this paper implements that the convolutional neural network for the classifications is also used for pretrained datasets. The preprocessing techniques are used for reducing the loss functions in entire image processing.

The article "Aerial Separation and Receiver Arrangements on Identifying Lung Syndromes Using the Artificial Neural Network" was published in 2022. Journal: Comput Intell Neurosci.

Toraman et al. [16] have implemented the novel artificial neural network approach to detect COVID-19 diseases from *X*-ray images using capsule networks; the image processing is one of the most crucial one to detect and prevent the diseases early; thus, this paper implements that the convolutional neural network helps to enhance the accuracy and the classification processes.

Kandaswamy et al. [17] have implemented the neural classifications of lung sounds using wavelet coefficient; this paper implements the accuracy classifications based on feature extraction and the configuration of the co-occurrence, the artificial neural network for the further classifications of the images, and the feature extraction technique are handled by the discrete wavelet transform.

Vardhana et al.[18] have implemented the convolutional neural network for biomedical image segmentation using hardware acceleration; artificial intelligence is one of the main concepts in the image processing systems; the feature extraction technique is handled by using the edge detection; thus, this paper shows that power is one of most important dominant features in image processing; the Sobel and the Prewitt algorithms play an important role in the entire network.

Varela-Santos and Melin [19] have implemented the new modular approach with fuzzy response integration for lung disease classifications based on multiple objective feature optimization in chest *X*-rays; this paper implements the hybrid approach for the modular artificial neural network, the classifications of the given datasets, and the feature extraction can be gathered by using the grey level co-occurrence matrixes and the local binary pattern; thus, the main features can be extracted by using the genetic algorithm.

Strzelecki and Badura [20] have implemented machine learning for biomedical applications. This paper proposed the classifications of the various types of algorithms and techniques used in medical image processing; artificial intelligence plays a vital role in the form of the support vector machine; thus, various types of feature extraction can be used in the image processing system.

Uguz [21] has implemented a biomedical system based on the artificial neural network and principal component analysis for the diagnosis of heart valve diseases. This paper implements the comparison of the image processing in the calculation of the heartbeat rate through listeners and the stethoscope; both are used in the efficient level but they could not predict more number of data collection; they have some limits for the calculations of the sounds establishment; thus, this paper implements the artificial neural network for the classifications of the given datasets and the feature extraction technique using discrete Fourier transform, and the feature reduction is detected by using the PCA technique.

The article "Aerial Separation and Receiver Arrangements on Identifying Lung Syndromes Using the Artificial Neural Network" was published in 2022. Journal: Comput Intell Neurosci.

Gao et al. [22] have implemented the holistic classification of CT attenuation patterns for interstitial lung diseases via a deep convolutional neural network. The entire difference of this paper provides holistic images in the dataset collections, which are gathered from the CT images. In the case of cardiac diseases, early detection and prevention are more crucial. Thus, this paper implements that the convolutional neural network for the classification of the images and the region of interest are used to detect the feature extraction. Thus, this technique will provide better accuracy and classification results in the image processing system.

Borwankar et al. [23] have implemented the improvised approach for respiratory pathologies classification with a multilayer convolutional neural network; this paper enhanced the hybrid approach for the entire network; thus, this paper implements the convolutional neural network for the classifications of the given datasets.

Zemouri et al. [24] have implemented deep learning in biomedical applications. This paper implies that the deep neural network is more effective than the support vector machine; thus, this paper shows that the different sets of datasets in the entire collection and the classification techniques take place through the convolutional neural network.

Anthimopoulos et al. [25] have implemented the lungs pattern classification for interstitial lung diseases using a deep convolutional neural network; this paper proposed that the computer-aided diagnosis using interstitial lung diseases (ILD) is classified by using the convolutional neural network, and thus the feature extraction function takes place. The effective classification consists of five networks, such as the RELU and the Max pool convoluting layer.

Wilson and Baietto [26] have implemented the advances in electronic-nose technologies developed in biomedical applications; this paper examines the biomedical applications in the medical field and a plenty of techniques and algorithms are detailed clearly, and the feature extraction of the image processing is detailed clearly; and finally, this paper compares the existing approach.

Pang et al. [27] have implemented a novel end-to-end classifier using domain transferred deep convolutional neural networks for biomedical images; this paper implements the dimensional reduction features using the distant deep neural networks, the classification techniques are handled by using the artificial neural network, and the datasets are pretrained by using the artificial neural network. Thus, this paper provides the enhanced accuracy when compared to the existing techniques.

The article "Aerial Separation and Receiver Arrangements on Identifying Lung Syndromes Using the Artificial Neural Network" was published in 2022. Journal: Comput Intell Neurosci.

Bullock et al. [28] have implemented the convolutional neural network (CNN) implementation for medical *X*-ray image segmentation, suitable for the small datasets in medical imaging; this paper implements the machine learning techniques for the classification of the lung images; the datasets collections are gathered from the *X*-rays and the comparison of this approach with the existing approaches, namely, clustering and entropy approaches.

Reddy and Rana [29] have implemented the biomedical image classifications using deep convolutional neural networks in overview; this paper implies that deep learning is much more efficient than machine learning (many existing papers compared and proven it); thus, this paper shows that deep neural network in the convolutional basis provides the enhanced output.

Demir et al. [30] have implemented the convolutional neural network-based efficient approach for the classifications of the lung diseases; this paper implies that the comparison of the two model approaches are used in the classifications of the accuracy. The first model is formed in the way of the convolutional neural network for the classifications, and the feature extraction is handled by using the SVM methods; then, the second phase consists of the classified neural approaches with the transfer learning methods. Commonly, the lung disease sounds are classified by using the short-term discrete Fourier transform (SDFT).

Cardenas et al. [31] have implemented the automated radiographic bone suppression with deep convolutional neural networks; this paper proposed that the 35 data sampled images are further divided into two phases, where 28 images are considered as the trained datasets and the balanced images are considered as the tested datasets; then, the feature extraction techniques take place in the form of data augmentation and the classifications techniques are handled by using the convolutional neural network. Thus, it provides better accuracy when compared to the existing techniques.

Jeya Jothi et al. [1] have implemented a comprehensive review of computational models for obstructive sleep apnea detection in biomedical applications. This paper proposed that diseases such as obstructive sleep apnea (OSA) are caused in the form of depression and mental disorder; therefore, this paper implements the various methods of preprocessing, feature extraction, segmentation, and classification techniques. Thus, the final results provide an enhanced output when compared to the existing techniques.

The article "Aerial Separation and Receiver Arrangements on Identifying Lung Syndromes Using the Artificial Neural Network" was published in 2022. Journal: Comput Intell Neurosci.

Sharma et al. [6] have implemented the novel fusion based on the convolutional neural network approach for the classifications of COVID-19 from chest *X*-Rays. COVID-19 is one of the most harmful diseases nowadays; this diseases mostly attack the lungs region in the form of the inhale and the exhale function and thus, early detection and prevention in image classification of the image processing are crucial ones; thus, this paper implements the convolutional neural network for the classifications functions using the VGG16 datasets.

Togacar et al. [3] have implemented the detection of lung cancer on chest CT images using minimum redundancy relevance feature selection methods with convolutional eural networks, and they have proposed that the AlexNet, LeNet, and the VGG16 datasets are used for the classifications of the convolutional neural network; this technique is commonly used for data augmentation techniques; it helps to reduce the dimensionality reduction and the cutting zooming process. Thus, it provides better accuracy when compared to the existing techniques.

### 1.2. Objectives

The main objective of the paper is to implement the accurate detection of the entire image processing. Thus, many existing algorithms provide the support vector machine and many techniques, but they could not predict better accuracy; thus, our paper implements the artificial neural network (ANN) for the classification technique, and the feature extraction is gathered by using the principal compound analysis technique. Thus, our paper provides an enhanced output when compared to the other existing techniques.

## 2. Overview of the Proposed Approach

The overview of the proposed approach explains the basic concepts of image processing.  Figure 1 implements that the overview of the proposed approach and the basic concepts of image processing are expressed clearly as the image processing techniques consist of the four major concepts, namely, preprocessing, segmentation, feature extraction, and classification techniques. The proposed artificial neural network provides enhanced results on the basis of feature extraction in image processing. Our proposed approaches imply the accuracy of classifications of lung diseases.

After the completion of feature extraction, the classification techniques take place. Our paper shows that the artificial neural network with the PCA methods is used to improve the classification accuracy when compared to the existing techniques.

The article "Aerial Separation and Receiver Arrangements on Identifying Lung Syndromes Using the Artificial Neural Network" was published in 2022. Journal: Comput Intell Neurosci.

### 2.1. System Model

The preprocessing technique is one of the important techniques in the image processing; the main function of the preprocessing technique is to help reduce the noise in the images and also enhance the RGB to the grey scale conversion in the images. In our proposed method, a Gaussian filter is used for removing the noise in the images.

The Gaussian filter is nothing but a low-pass filter, which helps to reduce the noise in the filter and also helps to reduce the blurred images. It helps to enhance the quality of the images; thus, the output of the Gaussian images helps to easily enhance the feature extraction processes.

(1) $$\begin{array}{c} G\left(x\right)=\frac{1}{\sqrt{2}*3.14\left(\alpha^{2}\right)}e^{y},\\ y=\frac{x^{2}}{2\sigma^{2}}. \end{array}$$

The above equation shows Gaussian functions of image processing.

#### 2.1.1. Particle Compound Analysis

Normally, feature extraction is used to extract the given dataset images into a group of manageable images, and then, this provides better-enhanced results when compared to the other existing techniques [8]. This paper shows that feature extraction is used for both dimensional reduction and the feature reduction process. It enhances the quality of the images and reduces the blurring in the image. This paper implements the conditions of

(2) $$\begin{array}{c} P\leq \mathrm{m,} \end{array}$$

where *P* is considered as the number of the significant principal components and *m* is considered as all the principal components. The above conditions imply that the principle compound analysis is used for the dimensional reduction, or it provides the lower dimensional in the entire image processing system. Let us assume that the datasets *Y* and *P* are considered as the principal compound analyses and *T* is considered as the covariance of the eigenvectors,

(3) $$\begin{array}{c} 1\leq P\leq m. \end{array}$$

#### 2.1.2. Discrete Fourier Transform

Normally, the mathematical expression in image processing can be used for the conversion of the signals at the given frequency, accurately; thus, this paper implements the DFT for feature extraction. The stethoscope sounds are generated in various domains and at various frequencies; in the form of the DFT transform, they are transferred at the given signal separately.

Thus, this function helps to predict the better accuracy of the classification obtained in this paper. Thus, the DFT transform does not give better results in the digital region. The form of medical image processing, especially in the lungs diseases classifications, provides enhanced accuracy classification results.

(4) $$\begin{array}{c} \;S_{r}=\sum_{K=0}^{N-1}X_{k\;}\text{Exp}\left(\frac{-2*3.14\mathrm{jrk}}{N}\right)\;r=0,\ldots ..N-1\text{,} \end{array}$$

where *n* denotes the number of samples and **S**_**r**_ denotes the DFT coefficient.  Figure 2 shows the proposed artificial neural network approach. The presented artificial neural network approaches demonstrate that the input data samples are preprocessed using the Gaussian filter. In the image processing technique, the Gaussian noise is introduced into the input images in the usual ways and is removed using the Gaussian filter. After the preprocessing procedures are finished, feature extraction techniques are used. In certain circumstances, feature reduction is regarded as the key idea, which lowers the need for dimensional reduction throughout the entire image processing process. Since feature extraction is the key idea, it reduces the dimensional spaces throughout all the photos and then offers image sharpening and smoothing.

The article "Aerial Separation and Receiver Arrangements on Identifying Lung Syndromes Using the Artificial Neural Network" was published in 2022. Journal: Comput Intell Neurosci.

## 3. Datasets

Our proposed methods take the 120 subjected dataset that might be the training phase; thus, our paper implies that the datasets are collected from the stethoscope, the given datasets are preprocessed by using the Gaussian filter, and then the feature extraction can take place in the form of the discrete Fourier transform and the feature dimensions can take place in the form of the principal component analysis (PCA). Then, the classification techniques can be handled by using the enhanced artificial neural network (EANN).

### 3.1. Materials and Methods

Figure 3 implements the materials and methods in our proposed methods. The materials and methods in our proposed methods show that the stethoscope dataset is given as the input layer after the completion of the preprocessing technique.

Artificial neural network is considered as the simple technique when compared to the many other existing techniques; it is considered as the learning approach and provides the neural cells easily; thus, the classification output provides an enhanced results when the feature extraction obtained the better accuracy.

The artificial neural network consists of three types of layers, namely,

- Input layer
- Hidden layer
- Output layer

Figure 4 represents the enhanced artificial neural network. The results obtained from the feature extraction give the input for the enhanced artificial neural network (EANN). This network consists of the input layer, hidden layer, and output layer. The input layer gathers the input data from the outer world, and these data are collected and approved by the hidden layer; also, the hidden layer processes the interaction in the form of the data collection in the entire image processing. After the completion process, this data is given through the input of the output layer [21].

(5) $$\begin{array}{c} \text{Sensitivity}=\frac{\text{TP}}{\text{TP}+\text{FN}}*100,\\ \text{Specificity}=\frac{\text{TN}}{\text{TN}+\text{FP}}*100,\\ \text{Accuracy}=\frac{\text{TN}+\text{TP}}{\text{TN}+\text{TP}+\text{FN}+\text{FP}}*100,\\ \text{Index}=\text{Sensitivity}+\text{Specificity}-1\text{.} \end{array}$$

The above equation shows the sensitivity, specificity, accuracy, and the index obtained from the given datasets, respectively.

The article "Aerial Separation and Receiver Arrangements on Identifying Lung Syndromes Using the Artificial Neural Network" was published in 2022. Journal: Comput Intell Neurosci.

## 4. Results and Analysis

In this section, our paper compares the many other existing techniques and approaches like the SVM with the DFT, the SVM with the PCA, and the DFT with the ANN [21], as shown in Figures 5–8. Thus, our paper provides an enhanced output accuracy when compared to the existing techniques.  Figure 5 shows the analysis of accuracy in the SVM with the DFT.

Figure 6 shows the analysis of accuracy in the SVM with the PCA.

Figure 7 shows the analysis of accuracy in the SVM with the PCA and the ANN.

Figure 8 shows the analysis of accuracy in the SVM with the PCA and the EANN.

Thus, Figure 9 implies that the result shows that our proposed method provides an enhanced output when compared to the existing technique.

## 5. Conclusions and Future Work

This work implements an enhanced artificial neural network for the classification of lung diseases. In the preprocessing technique, the Gaussian filter is used to remove the noise in the filter and provide better picture quality. Next, feature extraction techniques can take place in the form of the discrete Fourier transform. It shows that the heartbeat sounds separate depending on the particular frequency, and the feature reduction takes place by the principal compound analysis, and finally, the classification techniques take place with the support of an enhanced artificial neural network. In the future, this work can be improved with the SVM for the feature extraction process and the EANN for classification models.

## Figures and Tables

**Figure 1:** Overview of the proposed approach.

**Figure 2:** Proposed ANN approach.

**Figure 3:** Materials and methods.

**Figure 4:** Enhanced artificial neural network.

**Figure 5:** Analysis of accuracy in the SVM with the DFT.

**Figure 6:** Analysis of accuracy in the SVM with the PCA.

**Figure 7:** Analysis of accuracy in the SVM with the PCA and the ANN.

**Figure 8:** Analysis of accuracy in the SVM with the PCA and the EANN.

**Figure 9:** Total comparison case studies.

## Data Availability

The datasets used and/or analyzed during the current study are available from the corresponding author on reasonable request.
